# Early and High-Accuracy Diagnosis of Parkinson's Disease: Outcomes of a New Model

**DOI:** 10.1155/2023/1493676

**Published:** 2023-06-02

**Authors:** Sajjad Amiri Doumari, Kamal Berahmand, M. J. Ebadi

**Affiliations:** ^1^Department of Mathematics and Computer Science, Sirjan University of Technology, Sirjan, Iran; ^2^Department of Information Technology and Communications, Azarbaijan Shahid Madani University, Tabriz, Iran; ^3^Department of Mathematics, Chabahar Maritime University, Chabahar, Iran

## Abstract

Parkinson's disease (PD) is one of the significant common neurological disorders of the current age that causes uncontrollable movements like shaking, stiffness, and difficulty. The early clinical diagnosis of this disease is essential for preventing the progression of PD. Hence, an innovative method is proposed here based on combining the crow search algorithm and decision tree (CSADT) for the early PD diagnosis. This approach is used on four crucial Parkinson's datasets, including meander, spiral, voice, and speech-Sakar. Using the presented method, PD is effectively diagnosed by evaluating each dataset's critical features and extracting the primary practical outcomes. The used algorithm was compared with other machine learning algorithms of k-nearest neighbor (KNN), support vector machine (SVM), naive Baye (NB), multilayer perceptron (MLP), decision tree (DT), random tree, logistic regression, support vector machine of radial base functions (SVM of RBFs), and combined classifier in terms of accuracy, recall, and combination measure F1. The analytical results emphasize the used algorithm's superiority over the other selected ones. The proposed model yields nearly 100% accuracy through various trials on the datasets. Notably, a high detection speed achieved the lowest detection time of 2.6 seconds. The main novelty of this paper is attributed to the accuracy of the presented PD diagnosis method, which is much higher than its counterparts.

## 1. Introduction

Nowadays, much attention has been devoted to Parkinson's disease (PD), a neurological disorder that has made a prodigious impression on people globally [1, 2]. PD is a neurodegenerative disorder attributed to the deterioration of dopamine-producing neurons in the substantia nigra of the human brain [3]. Early clinical diagnosis of this disease is critical for patients so that they can receive appropriate treatment and care. Also, treatments like levodopa or carbidopa are significantly effective when administered early in the disease [3]. The early detection of Parkinson's disease is essential for preventing deteriorating health. More than 60% of dopaminergic neurons, which cause symptoms of gradual dysfunction in their motor system, can be eliminated with the initial control of the disease. PD is attributed to dopamine in the brain cells, and people suffering from PD have trouble doing their routines [4]. Other disease progression symptoms in the advanced stages include continuous eye movements, irregular sleep, and loss of olfactory sense. Such symptoms require proper diagnosis with accurate tools, and proper treatments must be defined for the disease; proposing an accurate method for early diagnosis of PD is of great significance. Accordingly, much literature has devoted much attention to this issue [5]. The presented papers compete with each other in terms of accuracy, speed, and authenticity. The obtained outcomes need to be reliable compared to the empirical results. However, it is better to avoid additional experiments to reach a generic diagnosis approach. Also, it is essential to see what technology can be.

In recent years, metaheuristic algorithms have received much attention for solving the complicated problems of search, prediction, diagnosis, and discrete and continuous optimizations. Such algorithms have brought appropriate solutions for continuous optimization problems, while the mathematical methods have mainly failed to offer optimal solutions, as mentioned in [6]. Metaheuristic algorithms, a subbranch of artificial intelligence, have countless applications in medicine and treatment. The AI model has been significantly developed for detecting the presence and severity of PD, considering nocturnal breathing patterns [7]. An umbrella term used for defining the application of machine learning (ML) algorithms is AI in the healthcare industry, with remarkable capabilities for diagnosis technologies in medical services. Basically, AI offers an intelligent computer system like humans for solving complicated problems, but ML presents more accurate output as it enables machines to learn from data [8]. Actually, ML employs mathematical data models to help a computer learn regardless of direct instruction. ML techniques contribute to analyzing the PD symptoms for early diagnosis and timely treatment of the disease [9, 10]. The significant drawback of PD diagnosis or other diseases is the high number of features and medical datasets that reduce accuracy, speed, and efficiency. In order to tackle such problems, metaheuristic algorithms can be used, and the optimization methods employed here play a key role in reaching this aim [11, 12]. Besides considering feature selection issues as an optimization problem, using metaheuristic algorithms is a promising technique for enhancing diagnosis accuracy [6].

The competition between the previous studies for presenting the most accurate PD diagnosis method using metaheuristic algorithms continues. Hence, the present paper is aimed at winning this competition by presenting an innovative model, namely, the crow search algorithm and decision tree (CSADT), for early PD diagnosis. The proposed model operates on four crucial PD datasets, including meander, spiral, voice, and speech-Sakar evaluating each dataset's critical features. CSADT is expected to have better results than other machine learning algorithms. Thus, the major innovation of this paper only lies in the heart of the diagnostic accuracy of the proposed method, which outperforms other state-of-the-art ones. Notably, studies have yet to yield this research's results. Also, the detection speed of this model is regarded as another novelty that competes with other related research. The main contributions of the paper are as follows:

- Combining crow search and decision tree algorithms (CSADT) for PD early diagnosis
- Implementing CSADT on four crucial Parkinson datasets, including meander, spiral, voice, and speech-Sakar, to evaluate each dataset's critical features
- Presenting high accuracy on the datasets

The rest of the paper is structured as follows: the previous work on using machine learning algorithms for PD prediction and detection is reviewed in the second section to highlight their significant gaps and shortcomings.  Section 3 presents the preliminary details of the crow search algorithm and the details of data preprocessing, data normalization, and so forth for the proposed method. In Section 4, the implementation results of the proposed method are presented according to valid Parkinson datasets. Finally, Section 5 provides conclusions and suggestions for future work.

## 2. Related Work

Many existing studies in the broader literature have examined the issue of PD diagnosis using various methods. In 2015, Shamir et al. addressed the issue of enlightening the course of treatment for Parkinson's disease by employing machine learning [13]. The combined form of support vector machine (SVM) [14], naïve Bayes (NBs) [15], and random forest (RF) [16] algorithms was presented to improve the PD treatment period. The empirical results indicated that the combination of NBs, SVM, and RF classifiers attained an accuracy of 86%. Besides, in 2016, Prashanth et al. scrutinized the accuracy of PD diagnosis using machine learning for feature extraction [10]. The authors demonstrated that among these three classification algorithms, SVM achieved an unsurpassed level of performance with 96% accuracy. In 2018, Mostafa et al. presented three important classifiers for PD diagnosis [17], in which multilayer perceptron (MLP) and decision tree (DT) [18] were considered. The authors aimed to analyze each classifier algorithm independently of its performance. The results obtained on numerous trials indicated that 91.63% and 91.01% of the highest accuracies belonged to the decision tree and multilayer perceptron, respectively, while the NBs algorithm had the lowest accuracy (89%). In 2018, Gupta et al. investigated the cuttlefish algorithm for diagnosing PD [11]. An improved cuttlefish recovery algorithm-based feature extraction method was developed. Comparing classifier algorithms within the decision tree and k-nearest neighbor (KNN) [19], the highest accuracy of 92% was obtained for the proposed optimized cuttlefish algorithm (OCFA). In 2018, Mostafa et al. evaluated several methods for diagnosing PD by classifying features [20]. Implementing five different algorithms of SVM, RFs, neural network (NN), NBs, and DT, a novel multiple feature evaluation approach (MFEA) was obtained for diagnosing PD on a multiagent system. The 10-fold cross-validation technique was used to estimate the model performance. The average rates of improvement were observed in the diagnostic accuracy of SVM (9.13%), RFs (12.75%), NN (9.19%), NBs (15.22%), and DT (10.51%) classifiers. In another study, Parisi et al. [21] proposed a new hybrid feature-driven algorithm for PD prediction, classification, and detection. The features were selected using the multilayer perceptron (MLP) approach and then classified through the Lagrangian support vector machine (LSVM) classifier. The proposed MLP-LSVM model performed at 100% on the area under the receiver operating characteristic curve, with relatively faster convergence.

Studies of ML techniques for PD diagnosis are well documented, but it is also well acknowledged that the issue of accuracy has always been important. To mention a few, in 2019, Chen et al. studied the effect of machine learning on the clinical analysis of PD [12]. The new algorithm was employed to extract the thalamic part, and then, SVM was used to predict PD from clinical conditions. The empirical results indicated an accuracy of 95% for the method employed in the PD diagnosis. In a cutting-edge paper from 2020, Sahni et al. used a multilayer perceptron algorithm based on quantum particle swarm optimization (QPSO) to address the issue of PD diagnosis [22]. The proposed multilayer perceptron had three layers to distinguish patients from healthy people. The experimental results revealed 93% accuracy based on the proposed algorithm. In another study, Senturk examined the early diagnosis of PD using machine learning algorithms [23]. The utilized classifier algorithms were regression tree (RT), artificial multilayer perceptron, and SVM. SVM showed enhanced performance with an accuracy of 93% compared to other classifier algorithms. The authors [24] used serum samples from a clinically well-characterized longitudinally monitored Michael J Fox Foundation cohort of Parkinson's disease patients with and without the prevalent LRRK2 G2019S mutation. The authors [25] proposed an approach based on an artificial neural network system with a backpropagation algorithm to assist clinicians in detecting Parkinson's disease. In this paper, the N2A-SVM algorithm is proposed as a novel prediction approach for Parkinson's disease gene prediction [26]. N2A-SVM consisted of three parts: a network for extracting gene characteristics, a deep neural network for lowering dimensions, and a machine learning method for predicting Parkinson's disease genes. Another study proposed a unique deep learning-based method for diagnosing Parkinson's disease using medical imaging [27]. Deep Convolutional and Recurrent Neural Networks (DNNs) benefit from training on medical images such as magnetic resonance images (MRIs) and DAT scans.

A large number of existing studies in the broader literature have examined many ML and deep learning (DL) models for predicting PD [28]. In 2022, Singh et al. used various ML algorithms for predicting PD based on voice recordings, and the results were acceptable [29]. In another study, Varalakshmi et al. proposed hybrid models based on DL and ML for feature extraction and feature classification for diagnosing PD based on hand drawing [30]. Due to the obtained results, the accuracy, sensitivity, and specificity scores were, respectively, 98.45%, 99%, and 98%. In 2023, deep belief network (DBN) was combined with neurofuzzy techniques for diagnosing PD, considering an ensemble learning method with the capability of online learning based on large clinical datasets. In order to handle such a dataset, a clustering method, namely, expectation maximization (EM), was employed. Additionally, the electroencephalographic (EEG) signals were employed as biomarkers for assessing the performance of Hjorth features [31]. The authors used SVM, KNN, and RF based on a 5-fold cross-validation methodology for classification. Lu and Sorooshyari examined seven EEG features calculated at single or combined spectral bands in sleep-wake and found that they differentiated the midbrain substantia nigra pars compact (SNc) lesions [32]. Besides, Table 1 outlines more related studies conducted so far and compared the outcomes of such studies in terms of accuracy.

Furthermore, feature extraction increases the accuracy of learned models as the features are extracted from the input data. The dimensionality of the data is also reduced at this stage, leading to increased training and inference speeds. Many previous and ongoing studies have used local pattern transformation based on feature extraction. For instance, in 2019, Tuncer and Dogan introduced a new octopus as a multiple-pooling method according to feature extraction [43]. Employing the proposed octopus's method for the signal in the preprocessing, the output signal was generated. The previous studies used the features extracted from vocal disorders as a precursor for PD detection since the patients encounter vocal variations and impairments in the early stages of PD [39, 44, 45]. Accordingly, Hoq et al. combined two methods based on a support vector machine (SVM), principal component analysis (PCA), and a sparse autoencoder (SAE) for detecting PD patients according to their vocal features. In 2019, Xiong and Lu stated that the vocal features of PD have an impact on individuals considering complex computational models [46]. Considering the vocal patterns, the PD diagnosis was examined by employing ML techniques by Lahmiri and Shmuel in 2019 [47]. Considering the Bayesian optimization method, the parameters of the radial basis function kernel of the SVM classifier were optimized, and acceptable results were presented. A novel multiagent feature filter (MAFT) algorithm was presented in 2021 to select the best features from the voice dataset and achieve PD symptoms [48]. Using a hybrid model (HM) combined with the MAFT increases the general accuracy by 96.9% and reaches more acceptable results.

Despite the remarkable interest in this regard and many studies conducted regarding efficient PD diagnosis models, many gaps and shortcomings still need to be addressed. No study has mentioned the benefit of using speech signal processing algorithms for PD investigations. In the current study [49], various speech signal processing algorithms are employed to extract clinically valuable information for PD diagnosis. The derived features are input to learning algorithms to build dependable decision support systems. The authors apply the tunable Q-factor wavelet transforms (TQWT) to the voice signals of PD patients for feature extraction, which has a higher frequency resolution than the standard discrete wavelet transform. To our knowledge, such a resolution has been observed for the first time. The primary aim here is to present a system for early diagnosis of PD based on a combination of decision tree and crow search algorithms used for four primary datasets of PD. Its final aim is to extract the essential features and design a robust system for the early diagnosis of PD.

## 3. Proposed Method

This section gives the most crucial information about the problem and the method proposed to solve it.

### 3.1. Preliminaries

In this study, four scientifically valid Parkinson's disease (PD) datasets were used: speech-Sakar, voice, meander, and spiral. Each dataset has its unique features, as characterized in Table 1. The proposed method and other comparable algorithms in this research were run on Python software. They paralleled each other in terms of essential features such as accuracy, precision, and recall. In Table 2, the Istanbul University of Neurology illustrated and arranged the Speech-Sakar dataset of 188 patients. The examined patients consisted of 107 males and 81 females. The Voice database of 31 patients, which the University of Oxford organized, was also studied. A total of 23 Parkinson's patients were included in this dataset. The meander dataset consisted of a questionnaire form with 158 participants. The Spiral dataset was also developed at the Faculty of Medicine of Botucatu, São Paulo State University, Brazil. The four datasets are the most imperative and reliable datasets on PD being used by researchers worldwide. Overall, an innovative combined method, namely CAADT, is proposed for early diagnosis of PD based on crew search and decision tree algorithms using these four valid datasets (Figure 1).

The flowchart presented outlines the entire process that must be considered in order to achieve the desired results. Accordingly, the user data needs to be normalized in the first step. Then, the crow search algorithm process initiates, whose pseudocode and supplementary information are given in Figure 2 (reprinted from [54]) and the Appendix.

When the solutions are converted to binary mode, the sigmoid function process initiates by selecting the subfeatures. Accordingly, the reduced dataset consisting of test and training data is entered into the decision tree. The output obtained after this process is assessed to specify the novel crows. Then, the memory is updated based on the invalid results, which need to be considered in assessing the crows and solutions. Notably, the normalization process is conducted for speech, voice, meander, and spiral before implementing the proposed method.

It should be noted that the voice dataset is regarded as a creative common speech dataset that acoustically affects reverberant environments with strong labels and truth data for transcription, denoising, and speaker identification. The primary sources used for extracting the voice dataset are references [14, 15, 22], according to which the proposed method is compared with the other selected algorithms, namely, the traditional curve fitting algorithm (TCFA), optimized cuttlefish algorithm (OCFA), and decision tree (DT). Furthermore, the speech-Sakar dataset from reference [53] is used to make additional comparisons to demonstrate the validity of the proposed method.

### 3.2. Normalization

In this stage, data normalization was performed on four PD datasets: meander, spiral, voice, and speech-Sakar. Normalization was conducted on the full features of each dataset. One of the essential methods of normalization is standard normalization. In the proposed method, each feature was normalized in the interval between the minimum MinX and the maximum MaxX; then, this interval was turned into a new interval of [New MinX, New MaxX] based on Equation (1). Accordingly, each value of *V* in each feature was normalized to a new one. The equation below states that the terms are used to normalize the data. Hence, the obtained results are used as the selected dataset for analysis.

(1) $$\begin{array}{c} \text{NewValue}=\frac{V-\text{Min}X}{\text{Max}X-\text{Min}X}. \end{array}$$

### 3.3. Crow Search Algorithm

In the proposed combined method (CASDT), the crow search algorithm has been used to select the features whose general introduction is given here. The crow search algorithm is a population-based metainnovative algorithm developed by Askarzadeh [54] based on the basic concepts of life and how crows acquire food. The main principles of this algorithm are restricted as follows:

- Crows live in groups
- Crows remember where they have hidden their food
- Crows chase one another to steal each other's food
- Crows protect their store of food from being stolen

It is noteworthy that the primary reasons for using CSA are its simple implementation, fewer parameters, flexibility, and so on [55]. From the optimization point of view in [54], crows are considered search agents and the natural environment where they live in the search space. In this algorithm, it is assumed that a certain number of crows are in a *d*-dimensional environment where the number of crows is denoted by the variable *N*, and the position of each crow is shown in Equation (2) [54]:

(2) $$\begin{array}{c} x^{i,\text{iter}}=\left[x_{1}^{i,\text{iter}},x_{2}^{i,\text{iter}},\cdots ,x_{d}^{i,\text{iter}}\right], \end{array}$$

(3) $$\begin{array}{c} i=1,2,\cdots ,N;\text{iter}=1,2,\cdots ,{\text{iter}}_{\max}, \end{array}$$

where *i* represents the number of crows or the solution in a search space, and iter is the representative of the current generation of iterations. The location of a crow in the search space of *d* dimensions and the total number of iterations are, respectively, shown by *x*^*i*^, iter, and iter_max_ [54].

As indicated in Figure 3 (adapted from [54]), *r*_*i*_ is a random number with a uniform distribution between 0 and 1, and fl^*i*,iter^ represents the flight length of crow *i* with iter repetition. Figure 1 indicates the schematic of this mode and the effect of fl on searchability. Small values of fl result in local search, and large values result in global search. As Figure 3(a) shows, if the value of fl is chosen less than 1, the next position of crow *i* is on the dash between *x*^*i*,iter^ and *m*^*i*,iter^. According to Figure 3(b), if the value of fl is chosen to be greater than 1, the next position of crow *i* is on the dash, which may exceed *m*^*j*^. Moreover, each crow has a memory to keep information in hiding. In the current iteration, the location of the crow's hiding place is displayed by *m*_*i*,iter_. In reality, the best location is stored in the memory of each crow. After initializing the location of hiding places of all crows, crow *i* can follow another crow, such as crow *j*, to touch its hiding place in which the two cases shown in the equation occur. As regards Figure 3, in the first case, crow *j* does not know that crow *i* is chasing him. Then, crow *i* finds the hiding place of crow *j*. In this case, the new location of crow *i* is gotten as Equation (3). In the second case, crow *j* knows crow *i* is chasing him and thus deceives him by going to another random location in the search space [54].

(4) $$\begin{array}{c} x^{i,\text{iter}+1}=\left\{\begin{array}{c} x^{i,\text{iter}}+r_{i}\times {\text{fl}}^{i,\text{iter}}\left(m^{j,\text{iter}}-x^{i,\text{iter}}\right)\;r_{j}\geq {\text{AP}}_{j,\text{iter}}\\ \text{a random location otherwise} \end{array}.\right. \end{array}$$

In Equation (4), *r*_*i*_ refers to a random number with an equal distribution between zero and one, and fl^*j*,iter^ indicates the flight length of crow *j* in iter iteration. AP^*i*,iter^  indicates the probability that crow *i* became aware of iter iteration. In the first case, everything relies on the value of the parameter fl^*j*,iter^. Figure 3 shows this issue in [54] and the effect of fl^*j*,iter^ parameter on the search. Based on Figure 3, small values of fl lead to local searches in the vicinity of *x*^*i*^ and iter, while large values of fl lead to additional searches. Similar to other metaheuristic algorithms, this algorithm utilizes an awareness probability (*AP*) parameter to balance exploration and productivity. The crow search algorithm's implementation process is described in 8 steps.

#### 3.3.1. Crow Search Algorithm for Initialization of the Parameters and Definition of the Optimization Problem

The optimization problem is initially defined in this step, and quantitative and qualitative parameters are then fixed. Some of these parameters, such as the minimum value of each variable (*X*min) and the maximum value of each variable (*X*max) and the number of problem dimensions (*d*), are set according to the problem. The configurable parameters of the crow search algorithm, such as crow population size (*N*), the total number of iterations (itermix), flight length (fL), and awareness probability (AP), are fixed beforehand. In this algorithm, the initial response for intensification and diversification is related to the parameters of AP. Accordingly, CSA seeks to find the local area by reducing the AP value where the best answer is. Using low AP levels, the intensity is improved. The AP values are directly proportional to the probability of searching in the current good solution drop domain. Accordingly, CSA specifies the search space randomly and improves diversity by employing high AP values.

#### 3.3.2. Crow Search Algorithm for Initialization of Location and Memory of Crows

Based on the optimization made in step one, the location and memory of crows are arbitrarily initialized in this step. Each crow specifies a possible response to the problem, and *d* signifies the number of decision variables. Providing that in the first iteration, crows have no decomposition; they can hide their food in their original locations. The location and memory of crows can be, respectively, shown as Equations (5) and (6) [54]:

(5) $$\begin{array}{c} \text{Location of crows}=\left[\begin{array}{ccccc} X_{1,1} & X_{1,2} & \; & \; & X_{1,d}\\ X_{2,1} & X_{2,2} & \cdots & \cdots & X_{2,d}\\ \vdots & \vdots & \cdots & \cdots & \vdots \\ \vdots & \vdots & \vdots & \vdots & \vdots \\ X_{n,1} & X_{n,1} & \cdots & \cdots & X_{n,d} \end{array}\right], \end{array}$$

(6) $$\begin{array}{c} \text{Memory of crows}=\left[\begin{array}{ccccc} M_{1,1} & M_{1,2} & \; & \; & M_{1,d}\\ M_{2,1} & M_{2,2} & \cdots & \cdots & M_{2,d}\\ \vdots & \vdots & \cdots & \cdots & \vdots \\ \vdots & \vdots & \vdots & \vdots & \vdots \\ M_{n,1} & M_{n,1} & \cdots & \cdots & M_{n,d} \end{array}\right]. \end{array}$$

#### 3.3.3. Crow Search Algorithm for Evaluation of All Crows or Solutions

In this step, similar to other metaheuristic algorithms, each solution is directed at the objective function to evaluate its quality or suitability for the objective function.

#### 3.3.4. Crow Search Algorithm for Production of New Locations

At this step, all crows move to the new position using Equation (4). The primary process of the crow search algorithm will be accomplished truthfully in two cases. In the first case, crow *j* does not know it is being chased by crow *i*. In this case, crow *i* finds the food hiding place of crow *j*. Then, the new location of crow *i* is obtained as Equation (4). In the second case, unlike the first case, crow *j* knows crow *i* is chasing him. In this case, crow *j* deceives crow *i* by going to another random place in the search space, which corresponds to the case (otherwise) in Equation (4).

#### 3.3.5. Crow Search Algorithm for Reviewing New Locations

At this step, if the new location is feasible and conceivable for each crow, that crow updates its location. Otherwise, it remains in its current location and makes no change to produce a new location.

#### 3.3.6. Crow Search Algorithm for Evaluation of All Crows or Solutions of New Locations

Each new solution, like the previous one, is sent to the objective function to determine its quality or suitability.

#### 3.3.7. Crow Search Algorithm for Memory Update

At this step, the newly achieved solutions are compared with those in the crow's memory, and if they are improved, they should be replaced in memory. Subsequently, crows update their memory based on Equation (7) [54].

(7) $$\begin{array}{c} m^{i,\text{iter}}=\left\{\begin{array}{cc} x^{i,\text{iter}} & Ff\left(x^{i,\text{iter}}\right)>f\left(m^{i,\text{iter}}\right)\\ m^{i,\text{iter}} & \text{otherwise} \end{array}.\right. \end{array}$$

Based on Equation (7), the crow memory will be updated, in which *f*(.) denotes the value of the objective function.

#### 3.3.8. Crow Search Algorithm for Reviewing the End Criteria

Each metaheuristic algorithm ends with a definite number of iterations iter_max_. Otherwise, steps 4 to 7 are repeated in the algorithm to iter_max_.

### 3.4. Turning Solutions Using the Sigmoid Function

All the solutions obtained from the crow search algorithm are continuous and cannot be directly used to solve binary or feature selection issues. Using mathematical transfer functions to convert continuous space to discrete space is one solution. In this research, the sigmoid or S-shaped function has been used for this purpose, which is defined in

(8) $$\begin{array}{c} \text{Sigmoid}\left({\text{CSA}}_{i}^{d}\left(t\right)\right)=\frac{1}{1+{\text{e}}^{-{\text{CSA}}_{i}^{k}\left(t\right)}}. \end{array}$$

In Equation (8), CSA_*i*_^*d*^, the constant value of the *i*th solution, is implied in the memory of the crow search algorithm for the *d*th dimension in iteration *t*. The sigmoid function transmits all the solutions in the crow memory to the space between 0 and 1, as shown in Figure 4. The outcome of the sigmoid transfer function is in the continuous mode between 0 and 1 and could not be directly used to answer the feature selection problem, as shown in Figure 4. As a result, thresholds must be considered for turning continuous solutions into binary. This research uses a random threshold to turn the crow search algorithm solutions into the binary mode in

(9) $$\begin{array}{c} {\text{CSA}}_{i}^{d}\left(t+1\right)=\left\{\begin{array}{cc} 0 & \text{if }\mathrm{rand}<\text{sigmoid }\left({\text{CSA}}_{i}^{d}\left(t\right)\right)\\ 1 & \text{if }\mathrm{rand}\geq \text{sigmoid }\left({\text{CSA}}_{i}^{d}\left(t\right)\right) \end{array}.\right. \end{array}$$

In Equation (9), CSA_*i*_^*d*^  represents the location of the *i*th solution in the agricultural land fertility algorithm population for the *d*th dimension in iteration *t*. The rand also represents several types of uniform distribution between 0 and 1. Based on Figure 5, a solution is initially generated in the continuous space of the crow search algorithm. Then, it is located in the space between 0 and 1 using a sigmoid transfer function and finally turned to binary mode with a random threshold for the desired solution.

### 3.5. Objective Function

In this research, the objective function of feature selection for the proposed algorithm is defined in Equation (10). To explain the objective function of the feature selection issue, a classifier algorithm is needed. In this research, the decision tree algorithm is adopted as the classifier.

(10) $$\begin{array}{c} \text{Fitness}=\alpha \gamma_{R}\left(D\right)+\beta \frac{\left|R\right|}{\left|N\right|}, \end{array}$$

where *αγ*_*R*_(*D*), |*R*|, and |*N*| display the decision tree error rate, the selected subset's linearity by the crow search algorithm, and the total number of features in the dataset, respectively. The parameters *α* and *β*, respectively, denote the significance of the classification quality and the length of the subset.

The proposed combined method, CSADT, was appraised in terms of accuracy, precision, recall, and combination measure F1. Concerning four criteria, the proposed algorithm is equaled with KNNs, SVM, NBs, MLP, and DT in Python software. The four criteria are mathematically defined below:

(11) $$\begin{array}{c} \text{Accuracy}=\frac{\text{TP}+\text{TN}}{\text{TP}+\text{TN}+\text{FP}+\text{FN}},\\ \text{Precision}=\frac{\text{TP}}{\text{TP}+\text{FP}},\\ \text{Recall}=\frac{\text{TP}}{\text{TP}+\text{FN}},\\ \text{F}1-\text{Measure}=\frac{2*\text{Precision}*\text{Recall}}{\text{Precision}+\text{Recall}}. \end{array}$$

In the above equations, all four criteria of accuracy, precision, recall, and combination measure F1 are formulated, with samples of true positive (TP), true negative (TN), false positive (FP), and false-negative (FN). In Figure 5, the results obtained from the implementation of each proposed method and other algorithms are shown on the meander, spiral, voice, and speech-Sakar datasets in terms of accuracy.

## 4. Results and Discussion

This section discusses the results obtained from implementing the proposed method on the selected data. According to Figure 6, the proposed method outperformed other algorithms with 93% accuracy in the speech-Sakar and 100% accuracy in the spiral, meander, and voice datasets. Accordingly, the proposed combined method gives more accurate results with values of 0.93, 1, 1, and 1 for speech-Sakar, spiral, meander, and voice.

Based on the results in Figure 7, the proposed method outperforms other selected algorithms with 92% precision in the speech-Sakar and 100% in the spiral, meander, and voice datasets. The second rank belongs to the decision tree regarding spiral and meander, with 98% and 97% values, respectively. On the other hand, k-nearest neighbors outperform the decision tree in terms of speech-Sakar and voice with an accuracy of 83% and 89%, respectively. Overall, SVM performs poorly compared to the others in every aspect.

Concerning the results shown in Figure 7, the proposed method performs better than the other algorithms, with 88% recall in the speech-Sakar and 100% precision in the spiral, meander, and voice datasets.

Finally, the time of the proposed combined algorithm for early diagnosis of PD was studied and compared with other algorithms, as shown in Figure 8. Based on the obtained results, the proposed algorithm was able to detect PD early and in near-zero time in most datasets and even four times faster than the decision tree algorithm in the speech-Sakar dataset. The combined algorithm in this paper was compared with that in [11], which proposed a method based on the cuttlefish algorithm called OCFA.

The comparison of the proposed CSADT algorithm with the OCFA method is demonstrated in Table 3. Accordingly, the proposed algorithm has achieved 100% accuracy, precision, recall, and combination measure F1. In terms of time, it performed faster than other algorithms, which is proven as an early Parkinson's disease diagnosis system.

For further assessment, the combined algorithm (CSADT) proposed in this research was compared with other essential algorithms proposed in references [14, 15, 22] on the voice dataset (Table 4). The proposed combined algorithm (CSADT) was compared with the RF, KNNs, DT, MLP, PSO, and QPSO algorithms on the voice dataset. The proposed combined algorithm, CSADT, achieved 100% on all four criteria and performed better than all other algorithms. This is indicative of an early and accurate diagnosis of PD disease. For further experimentation and evaluation, the combined algorithm (CSADT) implemented on the speech-Sakar dataset was compared with that employed in [53] for accuracy and combination measure F1. As shown in Table 1, CSADT outperforms the other algorithms by the greatest distance. Using this method, the medical problems in PD diagnosis can be significantly solved. The voice dataset used here can be extended to evaluate more findings and reach more accurate results. Practical experiences will validate the obtained results, and the proposed method should be used after it has been clinically validated.

In [53], the dataset was divided into several classes based on features wholly designated in Table 5.

In addition, a comparison was made among different machine learning algorithms, such as NBs, logistic regression (LR), KNNs, MLP, RF, Linear SVM, SVM of radial base functions (RBFs), and combined classifiers (ensemble). The proposed combined algorithm (CSADT) was also compared with [53] on the speech-Sakar dataset for numerous subfeatures, as shown in Table 6. As can be seen, the performance of the proposed combined algorithm (CSADT) was higher than that of NBs, LR, KNNs, MLP, RF, Linear SVM, SVM of RBFs, and the combined classifier in all the subsets of the speech-Sakar dataset. Therefore, 90% and 84% accuracy were achieved in the respective subsets of the baseline and MFCC features.

Another experiment was carried out on the speech-Sakar dataset with all other features except MFCC and TQWT in [53], as shown in Table 7. As can be observed, the performance of the proposed combined algorithm (CSADT) is more productive than the other algorithms in all features of the speech-Sakar dataset. The proposed combined algorithm (CSADT) resulted in an accuracy of 88% for all features except TQWT, 84% accuracy for all features except MFCC, and 93% for all the features.

Due to the results obtained so far, the superiority of the proposed method over its counterparts presented in the literature has been proven. Many optimization methods, like cross-validation, could be used in this research instead of the presented method. CSA is a novel swarm intelligence algorithm recently extended to simulating the crow's behavior in storing additional food and retrieving it when necessary [55]. The main drawback of the cross-validation method is that its training algorithm needs to be run from scratch *k* times, and it takes *k* times as much calculation to make an assessment. In comparison, CSA does not have this limitation and performs better than cross-validation methods in terms of accuracy.

It should be noted that the priority here is not a real-time prediction and accuracy matters. Hence, in order to have a reliable and accurate prediction, it is necessary to rerun the proposed method on the new dataset. The significant benefits are the high accuracy, precision, recall, and combination measure F1 obtained for the proposed model. The importance of a correct diagnosis of Parkinson's disease outweighs the importance of real-time prediction in the medical field. Hence, the proposed model can be considered a practical solution and prediction tool for the experts aiming to diagnose Parkinson's disease properly and prevent its progression. The innovation of the proposed method is attributed to its striking accuracy, authenticity, and reliability. Clearly, the datasets employed in this research are limited, and more comprehensive data can be considered to observe different results. As a result, the main reason CSADT has 100% accuracy is that the data considered is limited. The results obtained for other datasets are expected to have an accuracy of 90-100%. Notably, the proposed method outperforms the other examined models, which also compete with the other state-of-the-art ones presented in the literature. The accuracy of the obtained results lies at the heart of the minor difference between the prediction and empirical results. The obtained accuracy may be reduced for the other dataset, categorized in more detail, and includes a range of varieties.

## 5. Conclusions

In summary, a model, namely, CSADT, was provided for the early diagnosis of Parkinson's disease (PD). The proposed method was tested on four key PD datasets: meander, spiral, voice, and speech-Sakar. In the beginning, the normalization process was performed for speech, voice, meander, and spiral before implementing the proposed technique. Then, the procedure of the CSA was considered to evaluate the suitable solutions. The novel locations were generated and examined for conversion to binary mode. After this process, the sigmoid function specifies the subfeatures for the test and training datasets. The decision tree updated the assessed novel crows to reach the final results. Additionally, the presented algorithm was compared with other machine learning algorithms such as KNNs, SVM, NBs, MLP, DT, random tree, LR, SVM of RBFs, and combined classifiers in terms of accuracy, precision, recall, and combination measure F1. Besides, numerous trials have confirmed the proposed combined algorithm's high accuracy and early detection. The model was accurate with nearly 100% accuracy and fast due to the short diagnostic time for the diagnosis of PD. Finally, the proposed combined algorithm can be better implemented for PD detection in the case of seconds and milliseconds. The innovation of the proposed method (CSADT) is attributed to its striking accuracy, authenticity, speed, and reliability compared to other state-of-the-art ones presented in the literature. The drawback of the proposed method is attributed to the need for more comparisons with the obtained results and empirical ones. Also, more algorithms can be employed to specify the best ones, and a lack of statistical analysis is essential. Future investigations are necessary to validate the kinds of conclusions that can be drawn from this study. Future studies can examine the novel architectures of convolutional neural networks (CNN) and other algorithms. Further attempts could prove beneficial to the literature. As mentioned before, the 100% accuracy of the proposed model is attributed to the dataset considered for the proposed method, which has no inconsistencies or noise. The model is expected to perform correctly even in the case of a dataset with noise, although the accuracy will no longer be 100%. In future studies, it is recommended to consider the dataset with some inconsistency and noise and select the current prediction model. Accordingly, a more efficient method with other optimizers can be proposed as another model, and the current one and the novel one can be compared as a significant contribution to the future. The proposed model can combine the MLP or RF with the crow search algorithm. Besides, the principle component analysis (PCA) technique is a good idea for eliminating noise from the dataset.

## Figures and Tables

**Figure 1:** Flowchart of the proposed process.

**Figure 2:** The pseudocode of the crow search algorithm (this figure is reprinted from [54]).

**Figure 3:** Search mechanism by the crow in two modes (fl < 1 and fl > 1) (this figure is adapted from [54]).

**Figure 4:** Schematic overview of the sigmoid transfer function.

**Figure 5:** The process of continuous mode to binary using the sigmoid transfer algorithm in the proposed method.

**Figure 6:** Results obtained from the comparison of the proposed algorithm with other comparative algorithms in terms of accuracy.

**Figure 7:** Results obtained from the comparison of the proposed algorithm with other comparative algorithms in terms of precision.

**Figure 8:** Comparison of the proposed algorithm with other comparative algorithms in terms of time ().

**Figure 9:** The required steps for solving the problem (this figure is reprinted from [57]).

**Table 1:** A summary of the previous studies.

No.	Year	Method	Metaheuristic algorithms/algorithms	Accuracy
1	2018 [33]	An enhanced fuzzy k-nearest neighbor (FKNN)	The chaotic bacterial foraging optimization with Gauss mutation (CBFO) approach with FKNN	96.97%
2	2018 [34]	Combination of cardiac (MIBG) and cerebral ^123^I-ioflupane SPECT	A dual imaging	94%
3	2021 [35]	Dissolved gas analysis (DGA)	An efficient teaching-learning-based optimization (TLBO)	88.86%
4	2021 [36]	An automated tunable Q wavelet transform (A-TQWT)	Support vector machine	98.56%
5	2020 [37]	A new chaos-based stochastic model	Kernel-based naïve Bayes (KNB) algorithm	90%
6	2019 [38]	Eighteen feature extraction techniques	Machine learning techniques	92.94%
7	2019 [39]	Random forest, k-nearest neighbor classifier, and decision tree espy	The modified grey wolf optimization (MGWO) algorithm	98.28%
8	2020 [40]	The unified Parkinson's disease rating scale (UPDRS) and principal component analysis (PCA)	A deep neural network (DNN) model based on the reduced input feature space of Parkinson's telemonitoring dataset	MAE, RMSE, and *R*^2^ values of 0.926, 1.422, and 0.970
9	2022 [41]	The deep convolution neural network (CNN) method and ZFNet architecture	ML technique	The higher accuracy of 7.6% compared to other DL methods
10	2022 [42]	A wrapper-based binary improved grey wolf optimizer (BIGWO) method	BIGWO-V1 and BIGWO-V2 algorithms	Better than GA, PSO, BBA, and MCS algorithms

**Table 2:** Important and valid Parkinson's datasets.

Dataset	Number of features	Number of classes	Number of samples	Ref.
Speech-Sakar	754	2	756	[49]
Voice	23	2	194	[50]
Spiral	15	2	264	[51]
Meander	15	2	264	[52]

**Table 3:** Comparison of the proposed algorithm with OCFA [11].

Dataset	Algorithm	Evaluation criteria				
		Accuracy	F1-score	Recall	Precision	Time (second)
Voice	TCFA [11]	0.92	—	—	—	2.6
	OCFA [11]	0.94	—	—	—	2.1
	KNN [11]	0.87	—	—	—	—
	DT [11]	0.84	—	—	—	—
	**CSADT**	**1.00**	**1.00**	**1.00**	**1.00**	**0.02**

Meander	TCFA [11]	0.88	—	—	—	1.3
	OCFA [11]	0.89	—	—	—	0.9
	KNN [11]	0.78	—	—	—	—
	DT [11]	0.79	—	—	—	—
	**CSADT**	**1.00**	**1.00**	**1.00**	**1.00**	**0.04**

Spiral	TCFA [11]	0.88	—	—	—	1.3
	OCFA [11]	0.89	—	—	—	1.1
	KNN [11]	0.82	—	—	—	—
	DT [11]	0.79	—	—	—	—
	**CSADT**	**1.00**	**1.00**	**1.00**	**1.00**	**0.05**

**Table 4:** Comparison of the proposed combined algorithm CSADT with [14, 15, 22] on the voice dataset.

Algorithm	Accuracy	F1-score	Recall	Precision	Ref.
RF	0.95	—	—	**—**	[56]
KNN	0.90	—	—	**—**	
DT	0.89	—	—	**—**	
CSADT	**1.00**	**1.00**	**1.00**	1.00	

MLP	0.91	—	—	**—**	[53]
NB	0.89	—	—	**—**	
DT	0.91	—	—	**—**	
CSADT	**1.00**	**1.00**	**1.00**	1.00	

QPSO	0.93	—	—	**—**	[22]
PSO	0.81	—	—	**—**	
CSADT	**1.00**	**1.00**	**1.00**	1.00	

**Table 5:** Segmentation of the speech-Sakar dataset based on the different features of [53].

Entry	Feature	Number
1	Baseline	26
2	Bandwidth + formant	8
3	Mel-frequency cepstral coefficients (MFCC)	84
4	Wavelet transform applied to F0	182
5	Vocal fold	22
6	Tunable Q-factor wavelet transform (TQWT)	432

**Table 6:** Comparison of the proposed combined algorithm CSADT with [53] on the different subfeatures.

Algorithm	Vocal fold		Bandwidth + formant		Wavelet features extracted from F0		MFCC		Baseline	
	F1	Accuracy	F1	Accuracy	F1	Accuracy	F1	Accuracy	F1	Accuracy
NB	0.70	0.69	0.69	0.74	0.71	0.72	0.58	0.56	0.55	0.53
LR	0.72	0.76	0.72	**0.77**	0.72	0.76	0.82	0.83	0.75	0.79
KNN	0.71	0.76	0.71	0.76	0.71	0.73	0.77	0.80	0.71	0.75
MLP	0.72	0.75	**0.73**	0.76	0.74	0.78	0.81	0.82	0.75	0.77
RF	0.74	0.77	0.71	0.75	**0.75**	0.77	0.80	0.83	0.75	0.77
SVM (linear)	0.68	0.76	0.64	0.75	0.69	0.75	0.80	0.81	0.72	0.77
SVM (RBF)	0.72	0.77	0.71	0.77	0.72	0.77	**0.83**	**0.84**	0.74	0.77
Ensemble	0.72	0.76	0.70	0.76	0.70	0.75	**0.83**	**0.84**	0.75	0.79
CSADT	**0.74**	**0.80**	0.68	**0.78**	0.75	**0.84**	0.79	**0.84**	**0.85**	**0.90**

**Table 7:** Comparison of the proposed combined algorithm CSADT with [53] speech-Sakar dataset with other features except for MFCC and TQWT.

Algorithm	All features except TQWT		All features except MFCC		All features	
	Accuracy	F1	Accuracy	F1	Accuracy	F1
NB	0.65	0.67	0.81	0.81	0.83	0.83
LR	0.81	0.79	0.83	0.82	0.85	0.84
KNN	0.82	0.79	0.84	0.82	0.85	0.82
MLP	0.83	0.81	0.81	0.80	0.84	0.83
RF	0.79	0.78	0.83	0.82	0.85	0.84
SVM (linear)	0.81	0.80	0.84	0.83	0.83	0.82
SVM (RBF)	0.83	0.81	0.83	0.81	0.86	0.84
Ensemble	0.81	0.80	0.85	0.84	0.85	0.84
CSADT	**0.88**	**0.85**	**0.89**	**0.85**	**0.93**	**0.90**

## Data Availability

The data is available upon request from the first author.

## Appendix

### The Stages of Implementation

More information needed to understand the implementation process of the proposed method is outlined in Figure 9 reprinted from [57].

In the beginning, the problem and its parameters are tuned. Then, the problem, decision variables, and limitations are presented. Evaluating the customizable CSA parameters flock size, the highest number of iterations, flight period, and AP are considered. After that, the crows' location and memory need to be reset. The viable problem solution is indicated by each crow as the number of selection factors is denoted by *d*. Since the crows do not have any experience in the initial iteration, it can be concluded that they have hidden their meals at their first position. The objective function is evaluated by calculating the quality of the crow's location and considering the selection variable values in the objective function. A novel position is created for crows, and the viability of a new viewpoint is investigated in the following. The fitness and objective function considered for the novel places are specified. According to the value of the objective function, the crows' memories are upgraded. Steps 4 until 7 are conducted unless the highest number of iterations is obtained.
